# Deep Learning-Based Diagnosis Method of Emergency Colorectal Pathology

**DOI:** 10.1155/2021/3927828

**Published:** 2021-11-19

**Authors:** Chen Wang, Ning Zhang

**Affiliations:** ^1^Pathology Department, Wuhan Hanyang Hospital, Wuhan, Hubei 430050, China; ^2^Emergency Medicine, Wuhan No. 1 Hospital, Wuhan, Hubei 430022, China

## Abstract

One of the most common malignant tumors of the digestive tract is emergency colorectal cancer. In recent years, both morbidity and mortality rates, particularly in our country, are getting higher and higher. At present, diagnosis of colorectal cancer, specifically in the emergency department of a hospital, is based on the doctor's pathological diagnosis, and it is heavily dependent on the doctor's clinical experience. The doctor's workload is heavy, and misdiagnosis events occur from time to time. Therefore, computer-aided diagnosis technology is desperately needed for colorectal pathological images to assist pathologists in reducing their workload, improve the efficiency of diagnosis, and eliminate misdiagnosis. To address these issues, a gland segmentation of emergency colorectal pathology images and diagnosis of benign and malignant pathology is presented in this paper. Initially, a multifeatured auxiliary diagnosis is designed to enable diagnosis of benign and malignant diagnosis of emergency colorectal pathology. The proposed algorithm constructs an SVM-enabled pathological diagnosis model which is based on contour, color, and texture features. Additionally, their combination is used for pathological benign and malignant pathological diagnosis of two types of data sets D1 (original pathological image dataset) and D2 (dataset that has undergone glandular segmentation) diagnosis. Experimental results show that the proposed pathological diagnosis model has higher diagnostic accuracy on D2. Among these datasets, SVM based on the multifeature fusion of contour and texture achieved the highest diagnostic accuracy rate, i.e., 83.75%, which confirms that traditional image processing methods have limitations. Diagnosing benign and malignant colorectal pathology in an emergency is more difficult and must be treated on a priority basis. Finally, an emergency colorectal pathology diagnosis method, which is based on deep convolutional neural networks such as CIFAR and VGG, is proposed. After configuring and training process of the two networks, trained CIFAR and VGG network models are applied to the diagnosis of both datasets, i.e., D1 and D2, respectively.

## 1. Introduction

According to the Global Cancer Report data, which was released by the International Cancer Institute, the number of new cancer cases and mortality rates in the world were increasing in 2012 whereas nearly half of the new cancer cases occurred in Asia and most of these were in China [1]. In China, cancer has increasingly become a major threatening factor for the health of Chinese residents [2]. The prevention and treatment of cancer have become key to reducing the number of new cancer cases and mortality in our country and, thus, accurate pathological diagnosis is among core issues. Nowadays, medical pathological diagnosis work is mainly carried out by pathologists using microscopes to read the pathological slices of patients. The pathologist's diagnosis first takes a 3-4 *μm* live sample from the patient's suspected tumor area through puncture or surgery and then stains the sample to make a glass section for the read.

Initially, every pathologist observes the stained living sample in a slice through a microscope and finds the region of interest (ROI) of the suspected tumor. Then, he observes the cell morphology and structure in the area with a high-power microscope to determine whether the tumor is benign or benign according to the obtained pathological information. The level of malignancy and its degree of malignancy will ultimately determine the patient's treatment plan. However, the artificial pathological diagnosis method has certain shortcomings. First of all, there are a huge number of cells in pathological slices, and the tissue structure is complicated. Observing slices through a microscope is a time-consuming task [3]. Secondly, a large number of studies have shown that, particularly for the same pathological section, due to differences in the clinical experience of different pathologists, the diagnosis results are divergent, and different conclusions are drawn [4, 5]. Therefore, a diagnostic system is needed to be developed that has the capacity to assist pathologists in diagnosis and analysis, reduce their workload, and improve the efficiency of diagnosis [6].

With the rapid development of digital pathology technology, Computer-Aided Diagnosis (CAD), which is a combination of computer image processing technology and digital pathology technology, is used to simulate the diagnosis process of pathologists and obtain quantitative analysis results of pathology images with an expected level of precision and accuracy. Technology that provides a reference for diagnosis and prognosis analysis, i.e., computer-aided diagnosis technology, has obvious advantages over manual pathological diagnosis. Computer automatic analysis is used to reduce the workload of the pathologists such that he has more energy to pay attention to the development of the patient's condition. Quantitative analysis results help reduce differences between pathologists and effectively avoid misdiagnosis and improper treatment. The purpose of computer-aided diagnosis is not to replace doctors or pathologists but to assist doctors and improve the efficiency of patient diagnosis and treatment process. In addition, computer analysis can provide additional prognostic information. Compared with traditional human visual pathological features, computer analysis can generate new features, which will eventually surpass traditional pathological features.

According to the latest data report of China's urban cancer, which was released by the National Cancer Center in 2017, the mortality rate of emergency colorectal cancer in large, medium, and small cities is 19.08%, 12.41%, and 9.04%, respectively. Additionally, these are in cancer mortality. Therefore, a computer-aided diagnosis technology of emergency colorectal pathology images is needed to be developed in order to assist pathologists, reduce their workload, and improve the efficiency and effectiveness of patient diagnosis.

A gland segmentation of emergency colorectal pathology images and diagnosis of benign and malignant pathology is presented in this paper. Initially, a multifeatured auxiliary diagnosis is designed to enable diagnosis of benign and malignant diagnosis of emergency colorectal pathology. The proposed algorithm constructs an SVM-enabled pathological diagnosis model which is based on contour, color, and texture features. Additionally, their combination is used for pathological benign and malignant pathological diagnosis of two types of data sets D1 (original pathological image dataset) and D2 (dataset that has undergone glandular segmentation) diagnosis.

The remaining paper is organized as follows. In the subsequent section, a brief review of the relevant literature is presented which is followed by the proposed deep learning-based model and its applications in assisting pathologists and doctors. In Section 4, experimental observations are presented, and finally, concluding remarks are given in Section 5.

## 2. Related Work

Early research on medical pathology images is traced back to the 1990s [7–9]. With the rapid development of digital pathology and computer-aided diagnosis technology, a large number of auxiliary diagnosis methods based on medical pathology images have been proposed [10–11]. The tissue segmentation of pathology is equivalent to the process of finding the region of interest in the diagnosis process of pathologists. This work can provide important basic information for diagnosis [12] and is key to assisted diagnosis. However, the structure of pathological images is complex and the information content is large, which puts forward higher requirements for the effectiveness and practicability of auxiliary diagnosis methods. According to the survey, these methods are mainly divided into two aspects: traditional image processing methods and deep learning methods. Different from traditional methods, deep learning is a method of discovering distributed feature representations of data by combining low-level features to form a more abstract high-level representation attribute category or feature. With the deepening of deep learning research, scholars' research goals have gradually changed from simple images to complex images and the complexity of pathological images fits this point.

In recent years, deep learning methods have been widely used to analyze pathological tissue images. Among these methods is the deep convolutional neural network. Cirean et al. [13] used deep convolutional neural networks to detect mitosis in breast pathological tissues. The phenomenon, the Softmax classifier, is trained by learning the high-level features of the image to realize the classification of each pixel. Their work won the ICPR (International Conference on Pattern Recognition, ICPR) 2012 mitosis detection competition. Xu et al. [14] used a deep convolutional neural network combined with a sliding window method to segment the epithelial and matrix regions in pathological images, and its segmentation effect was much higher than that of traditional machine learning methods. Similarly, sliding windows have a time-consuming problem. For this reason, Long et al. [15] proposed a fully convolutional network for semantic segmentation, which pointed out a new direction for the improvement of pathological image tissue segmentation methods. Spanhol et al. [16] used deep convolutional neural networks to learn the characteristics of breast cancer pathological images for pathological diagnosis of breast cancer and achieved results that surpass traditional machine learning methods. According to the application results of deep learning methods in pathological image analysis, stability and robustness of deep learning have great advantages in the processing of digital pathological images. Lu et al. [17] used the deep convolutional neural network SegNet in the gland segmentation of emergency colorectal pathology images. Due to its small amount of data, the data was not expanded before training, which resulted in the unsatisfactory effect of gland segmentation. Ronneberger et al. [18] proposed a deep convolutional neural network U-net for gland segmentation of emergency colorectal pathology images. This method achieved good segmentation results and was time-consuming. Kain et al. [19] applied two deep convolutional neural networks, Object-Net and Separator-Net, to gland segmentation and auxiliary diagnosis of emergency colorectal pathological images, and achieved very high segmentation results and diagnostic accuracy. We have observed that deep learning methods are primarily used in the auxiliary diagnosis of emergency colorectal pathology images.

## 3. Proposed Deep Learning-Based Diagnosis Method

This section describes how the proposed deep learning-based diagnosis method is effective in resolving the aforementioned issues which are tightly coupled with the traditional diagnosis methods. Additionally, how computer-aided design is useful in improving the accuracy and precision of results is discussed in detail as well.

### 3.1. Neural Network Model

A neural network is a mathematical model that simplifies and abstracts the operating principles of biological neural networks [20]. It uses network topology knowledge as the theoretical basis and uses a weighted directed graph to simulate the connection between neurons in the brain. In the next step, it simulates the brain's nervous system's processing mechanism for complex information. Neurons are the basic units of neural networks. The earliest neuron model is the “M-P neuron model,” proposed by McCulloch et al. [21] in 1943. This model simulates the working mechanism of brain neurons very well; thus, it has been used to this day. In this model, there are input signals from *n* other neurons, and the expression of these signals is represented by the weight *w* of the connections between neurons. The neuron sums the received input value according to a certain weight overlap and compares it with the current neuron threshold  *θ* and then expresses the output through the “activation function.” The output is expressed as

(1) $$\begin{array}{c} y=f\left(\sum_{i=1}^{n}w_{i}x_{i}-\theta \right). \end{array}$$

The ideal activation function is a step function, as shown in Figure 1 and equation (2), which maps the input value to “0” or “1.” Among these values, “0” corresponds to inhibiting neurons, and “1” corresponds to exciting neurons. However, the step function has the characteristics of discontinuity and nonsmooth curve. Therefore, the application of this function is less. Equation (3) is the expression of the Sigmoid function, which has the capacity to generate output variable based on input values in a larger range to the range of (0, 1), and the function is continuous. Thus, the Sigmoid function is often used as the activation function in actual neural networks.

(2) $$\begin{array}{c} \mathrm{sgn}\left(x\right)=\left\{\begin{array}{cc} 1, & x\geq 0,\\ 0, & x<0, \end{array}\right) \end{array}$$

(3) $$\begin{array}{c} \text{sigmoid}\left(x\right)=\frac{1}{1+e^{-x}}. \end{array}$$

The actual neural network structure is composed of countless “MP neurons” connected at a certain level, mainly including the input layer, hidden layer, and output layer. Among them, there can only be one input and output layer, and the hidden layer can have multiple.  Figure 2 shows a simple neural network structure diagram. Each layer of the structure is composed of multiple neurons, and each layer of neurons is fully connected to the next layer of neurons. Such a neural network structure is usually called a “multilayer feedforward neural network.” The learning process of the neural network is to adjust the weights between neurons and the threshold of each neuron according to the training data. Therefore, the information obtained in the learning process is contained in the connection weights and thresholds.

### 3.2. Deep Convolutional Neural Network

On the basis of traditional neural networks, Professor Hinton of the University of Toronto proposed the concept of deep learning [22]. The deep learning model extracts deeper features in the image through a sophisticated learning process of massive data and then achieves a better classification effect. Deep Belief Network [23], Autoencoder, Deep Convolutional Neural Network [24], etc., are among the commonly used deep learning models. The most commonly used is the deep convolutional neural network model. Deep convolutional neural networks are currently widely used in image recognition and classification. Its structural features of local connection and weight sharing reduce the complexity of the network model, reduce the number of parameters, and make it more similar to a biological neural network. It is the first learning algorithm to truly successfully train a multilayer network structure.

### 3.3. SegNet-Based Gland Segmentation Method for Emergency Colorectal Pathological Images

SegNet has an encoding network (Encoder) and a corresponding decoding network (Decoder). The network structure is symmetrically distributed, input is the input image, and output outputs the divided image. The coding network part includes 13 convolutional layers (Convolution), including batch normalization [25], Rectified Linear Unit [26], and pooling that cooperate with it; the decoding network includes the same 13-layer convolutional layer and corresponds to the pooling layer upsampling. The network finally classifies the pixels through the Softmax classifier to complete the segmentation.

In the encoding process, the input image is first convolved to obtain feature maps. After these feature maps are normalized by BN, they are activated by the element-level modified linear unit ReLU and then sent to the pooling layer for maximum pooling to complete downsampling; In the decoding process, the decoded feature map is obtained through upsampling, and then, the final feature map is obtained after convolution, normalization, and activation. The Softmax classifier is trained through the feature map so that the classifier can perform each pixel. Points are classified independently. SegNet is different from deep convolutional neural networks in that it uses a batch normalization layer (BN) and ReLU activation function.

#### 3.3.1. Introduction to Batch Normalization Layer

In a deep convolutional neural network, if the output of the activation function in the network is larger, then its learning gradient is smaller. Thus, the learning rate of the network is slower. This results in the deep convolutional neural network, the shallow layer is basically not learned, the weight change is small, the learning task is mainly in the last few layers of the network, and such a network loses the meaning of depth. The batch normalization layer is mainly used before the activation function, by normalizing the input of each layer to ensure the stability of the input data of each layer, so as to achieve the purpose of accelerating training. Batch normalization is to normalize the distribution of each layer of input data to a distribution with a mean of 0 and a variance of 1:

(4) $$\begin{array}{c} {\hat{x}}^{\left(k\right)}=\frac{x^{\left(k\right)}-E\left(x^{\left(k\right)}\right)}{\sqrt{\text{Var}\left(x^{k}\right)}}. \end{array}$$

Among these variables, *x*^(*k*)^ represents the *k*-th dimension of the input data, *E*(*x*^(*k*)^) represents the average value of the data in this dimension, and $\sqrt{\text{Var}\left(x^{k}\right)}$ represents the standard deviation of the input data in this dimension.

Although the data distribution of each layer is fixed after such processing, this distribution is not necessarily the distribution learned by the previous layer, so forcibly normalizing will destroy the learned features. Therefore, batch normalization is set in two learnable variables *γ* and *β*, and then, these two variables are used to restore the data distribution learned in the previous layer:

(5) $$\begin{array}{c} y^{\left(k\right)}=\gamma^{\left(k\right)}{\hat{x}}^{\left(k\right)}+\beta^{\left(k\right)}. \end{array}$$

In the network training process, the batch normalization layer restores the data input of the previous layer by adjusting *γ* and *β* and fixes the originally unfixed data distribution, thereby accelerating the network training.

#### 3.3.2. ReLU Activation Function

The activation function in the traditional neural network structure generally uses the Sigmoid system such as Logistic-Sigmoid and Tanh-Sigmoid. The mathematical expressions and graphs are as follows:

(6) $$\begin{array}{c} \text{Sigmoid}:f\left(x\right)=\frac{1}{1+e^{-x}}, \end{array}$$

(7) $$\begin{array}{c} \text{Tan}h:f\left(x\right)=\frac{e^{x}-e^{-x}}{e^{x}+e^{-x}}. \end{array}$$

We have observed that expressions and images in which Sigmoid and Tanh functions are the activation functions of the deep convolutional neural network have obvious defects; that is, these are both saturated nonlinear functions. The so-called saturation means that when the input reaches a certain value, the output no longer changes. This feature will block the transmission of part of the data, which is not conducive to network training. The emergence of ReLU and Softplus activation functions makes up for the shortcomings of the Sigmoid system activation function. Compared with Sigmoid and Tanh, ReLU and Softplus have a relatively wide excitation boundary, which is closer to the activation model of human brain neurons. From the expression and function curve, Softplus is regarded as the smoothness of ReLU. However, because ReLU has the characteristics of unilateral inhibition, this makes the output of some neurons be 0 during the training process, making the network sparse, thereby reducing the interdependence between parameters, which can reduce overfitting to a certain extent. However, Softplus does not have sparseness; therefore, the ReLU function is more in line with the actual activation model of biological neurons.

(8) $$\begin{array}{c} \text{ReLU}:f\left(x\right)=\max\left(0,x\right), \end{array}$$

(9) $$\begin{array}{c} \text{Softplus}:f\left(x\right)=\log\left(1+e^{x}\right). \end{array}$$

Therefore, an emergency colorectal pathology image data set and its expansion method are presented here to address these issues, specifically the problem of gland segmentation in emergency colorectal pathological images. The proposed model has provided a research method for the emergency diagnosis of colorectal pathology as described above.

## 4. Experiments and Discussions

This section briefly explains various experiments which were conducted to verify the exceptional performance of the proposed deep learning-based model. Additionally, it explains how the proposed model helps in assisting pathologists and doctors to improve the accuracy and precision ratio of various results.

### 4.1. CIFAR Network and VGG Network

(1) The CIFAR network is a deep convolutional network model proposed by Alex for the data set CIFAR-10. The network uses a simple network layer structure and has achieved high classification accuracy on the CIFAR-10 multiclass data set. We have observed that this network has good predictive performance. Therefore, this network is selected for the research of emergency colorectal pathology diagnosis in the proposed model.
From the network structure, CIFAR input is an image and output is a Softmax classifier. The network contains three layers of convolutional layers, 3 layers of pooling layers, and 1 fully connected layer. In addition, there are 3 activation function layers and 2 local response normalization layers (local response normalization, LRN).
The principle of local response normalization is to imitate the “side inhibition” phenomenon in the structure of biological neural networks; that is, activated neurons will inhibit the activation of neighboring neurons. The purpose of normalization here is to “inhibit,” where the local response normalization draws on the idea of “lateral inhibition,” and creates a competition mechanism for the activity of local neurons, making the response larger value relatively larger and improving the generalization of the model. *Ability*. The following formula is the formula for the normalized layer function of the local response:
  (10) $$\begin{array}{c} b_{x,y}^{i}=\frac{a_{x,y}^{i}}{{\left(k+\alpha \sum_{j=\max\left(0,i-\left(n/2\right)\right)}^{\min\left(N-1,i+\left(n/2\right)\right)}{\left(a_{x,y}^{j}\right)}^{2}\right)}^{\beta }}. \end{array}$$
(2) The VGG network [27] was proposed by Karen et al. in the 2014 ImageNet competition. This network model uses multiple small-size convolution kernels instead of large-size convolution kernels, which can reduce parameters on the one hand and is equivalent on the other hand. More nonlinear mapping has been performed to increase the fitting ability of the network model. The model won the championship in the competition that year. Therefore, this network is used for the research of colorectal pathological diagnosis.

The network structure is obtained, network input is an image, and output is a Softmax classifier. The network contains 13 convolutional layers, 3 pooling layers, 15 activation function ReLU, 3 fully connected layers, and 2 dropout layers, where each convolutional layer is followed by an activation function; the first two are fully connected layers followed by an activation function and a dropout layer.

### 4.2. Experimental Setup

The experimental platform is Linux system Ubuntu14.04, the processor is Intel Xeon (R) CPU E5-2620 v3 @2.40 GHz, the memory is 32 GB, the graphics card is Nvidia GeForce GTX 1080, the development environment is the Caffe framework, and the development language is Python2.7.6. Additionally, the development tool is Matlab R2014a. The support vector machine (SVM) classifier selects the Gaussian kernel LIBSVM and uses 100 10-fold cross-validation to determine the accuracy of the Gaussian kernel parameters. The experimental data set includes two types. (i) The first type is a data set expanded by the scale transformation, including 425 training sets and 400 test sets, called D1. (ii) The second type is a pathological image set that only retains the gland part after segmentation. The number of the training set and test set remains unchanged, called D2.

The purpose of the experiment is to compare auxiliary diagnosis effects of different depth convolutional neural networks in colorectal pathological images, and, on the other hand, to examine the influence of glandular segmentation from the perspective of colorectal pathological images auxiliary diagnosis. We intend to use CIFAR and VGG networks for training and auxiliary diagnosis tests on D1 and D2, respectively. CIFAR1 and CIFAR2 are used to represent the results of training and diagnostic testing of the CIFAR network on D1 and D2, respectively. Similarly, VGG1 and VGG2 represent the results of training and diagnostic testing of the VGG network in D1 and D2, respectively. In the training process of the CIFAR network, the basic learning rate base-lr is set to 0.001, the learning rate change rate lr-policy is set to “fixed,” the momentum is set to 0.9, the weight decay is set to 0.004, and the network model is saved every 1000 iterations. In order to improve the training effect of the network, the training process is accompanied by testing; you can set a fixed number of network iterations to test once and adjust the network parameters according to the testing effect. The number of test iterations test-iter is set to 5, and the test interval is set to 500. The basic learning rate base-lr of the VGG network during training is set to 0.003, the learning rate change rate lr-policy is set to “step,” the learning rate change index gamma is set to 0.1, the learning rate change frequency step size is set to 1000, and the momentum is set to 0.9. The weight decay is set to 0.0005, and the network model is saved every 1000 iterations. The number of test iterations test-iter is set to 40, and the test interval is set to 1000. When using the test set for diagnostic testing, the voting method in Section 4 is used to determine the benign and malignant of each pathological image.

### 4.3. Results and Analysis

For dataset D1, Figure 3 shows the training curves of CIFAR and VGG. It is evident from Figure 3 that the CIFA network gradually converges after 10000 iterations, and the VGG network gradually converges after 8000 iterations. The convergence speed of the VGG network is faster. In addition, the test accuracy of CIFAR is close to 0.95, the test accuracy of VGG is closer to 1, and the loss value of VGG is closer to 0 compared to CIFAR. Thus, the training effect of VGG is better. For dataset D2, Figure 4 shows the training curves of CIFAR and VGG. It is evident from Figure 4 that the CIFAR network starts to converge around 10,000 iterations, and the VGG network also starts to converge around 10,000 iterations. The convergence speeds of the two are equivalent. However, the test accuracy of the VGG network is higher than that of CIFAR, the loss value is also lower, and the curve trend is stable, so VGG has achieved a better training effect. When using the test set for diagnostic testing, for dataset D1, the CIFAR network model with 15,000 iterations and the VGG network model with 10,000 iterations are selected for testing. For dataset D2, a network model with 10,000 iterations was selected for testing. The diagnostic test results of the two networks in the two types of data sets and the results of other methods are shown in Table 1, and the diagnostic ROC curves of the two networks are shown in Figure 5.

It can be seen from the data in the table that the overall diagnostic effect of CIFAR and VGG in D2 is higher than the result in dataset D1. It can be seen that segmenting the gland structure can effectively improve the accuracy of pathological diagnosis. In addition, the overall diagnostic accuracy of the VGG network is higher than that of the CIFAR network, which shows that VGG has a better pathological diagnosis effect. In addition, the diagnostic accuracy of this chapter is significantly higher than that of the diagnosis method under the multifeature description in Chapter 4, which shows that the deep learning method has obvious advantages in auxiliary diagnosis. In order to compare the effects of the methods in this chapter, the pathological diagnosis results of the other two methods are listed in the table, based on SegNet and Object-Net, respectively.

For the TPR, the diagnostic accuracy of VGG in D1 is 2.7% higher than the result of CIFAR, and in D2, the diagnostic accuracy of VGG is 5.41% higher than the result of CIFAR, which further verifies the segmentation of glands. The effect of rediagnosis is better. In the other two networks, SegNet is not very effective in diagnosing benign pathology, with an accuracy rate of only 54.5% and almost no diagnostic effect. The Object-Net's benign accuracy rate reached 97.29%. Among 37 benign pathological images, only one image was diagnosed as malignant. In comparison, the best result of the method proposed in this chapter is 94.6%. Among the 37 benign pathological images, it is equivalent to 35 correctly diagnosed, and good diagnostic results have also been achieved.

For TNR, the diagnostic accuracy of VGG in D1 is 2.32% higher than that of CIFAR. On D2, CIFAR has achieved 100% diagnostic accuracy, while the result of VGG is slightly lower than that of CIFAR. In addition, the diagnostic accuracy of SegNet in malignant pathological images has reached 100%, and the results of Object-Net are the same as VGG2, which is 96.67%, which is equivalent to 42 of the 43 malignant pathological images correctly diagnosed. Apart from it, only 1 Zhang made a wrong diagnosis, and the overall diagnosis effects are good.

For the overall diagnostic accuracy rate of ACC, in the two data sets, the diagnostic effect of VGG is higher than that of CIFAR. Combined with the ROC curve in Figure 6, the diagnostic ROC curve of VGG in the two types of data sets is higher than that of CIFAR. It is more inclined to the upper left corner of the coordinate, and the corresponding AUC value is also higher. Among them, the AUC value of VGG on D2 is 0.9768, which is higher than the other results, which is consistent with the results of diagnostic accuracy. Judging the diagnosis results of the other two networks, SegNet's diagnostic accuracy rate is low, and the diagnosis effect is poor. Object-Net achieved the highest diagnostic accuracy rate of 97.5%, which is equivalent to 78 pathological images correctly diagnosed in the 80 test set. In contrast, in the method proposed in this paper, the highest diagnostic accuracy rate is 96.25%, which is equivalent to 77 pathological images that have been correctly diagnosed, and good diagnostic results have also been achieved.

Although the VGG network has achieved good diagnostic results, it is still not the best. The reason is that, on the one hand, the colorectal pathology image is complex and difficult to diagnose; on the other hand, because this chapter mainly does configuration work in the application of the network, the structure of the network and its parameters have not been adjusted too much. The network can be optimized by adjusting the network structure or specific layer parameters to obtain a higher diagnostic effect. Finally, through experimental comparison and analysis, the diagnostic accuracy rate of the VGG network is higher than that of the CIFAR network and the diagnosis effect is better.

## 5. Conclusion and Future Directions

In the diagnosis process of emergency colorectal cancer, the diagnosis method of pathologists is not only time-consuming and highly subjective but also easy to cause misdiagnosis events, which is very unfavorable to the treatment of patients. Therefore, there is an urgent need to study the computer-aided diagnosis technology of colorectal pathological images to provide doctors with accurate auxiliary analysis results along with speeding up the treatment process. To address these problems of emergency colorectal pathological diagnosis, a deep learning-based hybrid method, which is based on gland segmentation method and two pathological diagnosis methods, is presented. The main contributions of this paper are as follows. (1) A detailed investigation, analysis, and evaluation of the domestic and foreign research status of auxiliary diagnosis methods which are based on traditional image processing and deep learning-based auxiliary diagnosis methods are made. (2) The theoretical contents of the neural network and deep convolutional neural network are introduced. (3) A method of gland segmentation based on SegNet-based colorectal pathological images is proposed. First, the colorectal pathology image data set Warwick-QU was expanded. Then, we configure and train the SegNet network structure. (4) A colorectal pathology-assisted diagnosis method based on deep learning is proposed. The network model is obtained by configuring and training two deep convolutional neural network models CIFAR and VGG, and the network model of the trained network is used to assist in the diagnosis of pathological images. Finally, a comparative analysis of the auxiliary diagnosis results through the diagnosis indicators shows that the diagnosis effect of CIFAR and VGG is much higher than the diagnosis effect of SVM based on contour and texture features. In these two networks, the diagnostic effect of VGG is better than that of CIFAR.

In the future, we have planned to implement the proposed scheme in the real environment of hospitals where we will practically observe how the proposed scheme is effective in resolving the aforementioned issue and assisting pathologists.

## Figures and Tables

**Figure 1:** M-P Neuron model.

**Figure 2:** Multilayer feedforward neural network.

**Figure 3:** CIFAR training curve in dataset D1.

**Figure 4:** VGG training curve in dataset D1.

**Figure 5:** CIFAR training curve in dataset D2.

**Figure 6:** VGG training curve in dataset D2.

**Table 1:** Diagnosis results of different methods in datasets D1 and D2.

Data set	Method	TPR (%)	FPR (%)	TNR (%)	FNR (%)	ACC (%)
D1	CIFAR1	89.19	10.81	90.7	9.3	90
	VGG1	91.89	8.11	93.02	6.98	92.5

D2	CIFAR2	89.19	10.81	100	0	94
	VGG2	94.6	5.4	97.67	2.33	96.25

Warwick -QU	SegNet	54.5	45.5	100	0	73.7
	Object-Net	97.29	2.71	97.67	2.33	97.5

## Data Availability

The datasets used and analyzed during the current study are available from the corresponding author upon reasonable request.
